# Comparison of the Meta-Active Machine Learning Model Applied to Biological Data-Driven Experiments with Other Models

**DOI:** 10.1155/2021/8014850

**Published:** 2021-12-13

**Authors:** Hao Wang

**Affiliations:** State Grid Electric Power Research Institute, Beijing, China

## Abstract

Currently, many methods that could estimate the effects of conditions on a given biological target require either strong modelling assumptions or separate screens. Traditionally, many conditions and targets, without doing all possible experiments, could be achieved by driven experimentation or several mathematical methods, especially conversational machine learning methods. However, these methods still could not avoid and replace manual labels completely. This paper presented a meta-active machine learning method to resolve this problem. This project has used nine traditional machine learning methods to compare their accuracy and running time. In addition, this paper analyzes the meta-active machine learning method (MAML) compared with a classical screening method and progressive experiments. The obtained results show that applying this method yields the best experimental results on the current dataset.

## 1. Introduction

Nowadays, thousands of data-driven experiments are carried out not only in academia but also in industry. For this, relevant algorithms have been modified; as a result, biological experiments have been improved [1, 2]. This improvement is because these experiments are usually performed manually or sometimes through simulation experiments, avoiding the moral, social, and waste of resources problems that actual biological experiments could probably cause. Traditional machine learning methods are convenient to calculate the relationship between independent and dependent variables in big data under rules [3, 4]. However, it is difficult to conceive rules, determine categories, and label in most practical applications. For example, the nearest neighbour method is used to cluster drug and clone datasets about 30 rounds [5]. Active machine learning methods significantly reduce the labelling workload by manual [6]; however, it still requires people to label complex samples [7]. The built model can no longer be used for other rules or situations [8]. The process will try to compare pool-based active learning based on the SVM or decision tree method with the classical one [9].

The inputs of meta-active learning methods are no longer just different data but different tasks. Therefore, these methods could satisfy many applications of few-shot learning and maximize the universal ability of their models [10]. In addition, metalearning methods directly learn parameters in the loss function. The parameter model learned from different tasks depends on [11]. For instance, MAML only focuses on initialization parameter [12]; this method is used to initialize parameters and then see the effect on different tasks. In other words, let the machine learn the learning algorithm. In a nutshell, learn to learn.

The paramount significance of this study is that, in actual biological experiments on protein compound effects, a large number of professionals are inevitably required to invest in the experiments to determine the validity of the experimental results manually. This article firstly uses experiments to prove that traditional machine learning can reduce manual screening experiments. However, the accuracy of the model is very dependent on a large number of manually accurate labels. Therefore, this project tries various commonly used machine learning methods to build models, even the optimized models. Then, this article uses experiments to further prove that meta-active learning can be compared and proved by the actual accuracy. Under the premise of few artificial labeling, the performance related to the previous experiment provides references and methods verification. The concept graph is shown in Figure 1.

## 2. Overview

The overview of this article could be divided into three levels: dataset level, model level, and verification level, as shown in Figure 2.

The data input used in the three main machine learning experiments is derived from the same data source at the model level. However, the input is a different part of the split data source. At the same time, in order to consider the characteristics of the model more comprehensively, the method of verifying the optimal model is also completely different. After each step of the experiment has been completed, the best model will transition from the reasonable optimal model of the previous experiment to the next experiment. Then, it is used to compare further and judge the better model.

## 3. Methods and Experiments

This section briefly discusses the experimental steps, dataset analysis, model design, and meta-active learning (MAML) designed.

### 3.1. Experimental Steps

The experiment of this paper is conducted using the following four steps:

Step 1: data preparation:
(i) Mainly, the work collates phenotypes' data in round 1–30 and turns them to true or false
  Original data are the score for nodes that are computed by measuring the average performance of a 1-nearest neighbour classifier
  True (1) means this score of the cluster is highly probably correct
  False (0) means this score of the cluster is highly probably incorrect
(ii) Find out which is the independent (y_label) and dependent (x_feature) variables
(iii) Do some necessary calculations, such as mean and variance
  Step 2: traditional machine learning methods:
  When training models, this experiment will use 80% as the training dataset and 20% as the test dataset
  After that, this project will describe classifier errors by accuracy and time
  Step 3: meta-active learning methods:
  Pool-enabled active learning based on logistic regression with normalization and loss function
  MAML method focuses on the initialization parameter
Step 4: make a conclusion:
  The receiver operating characteristic (ROC) analysis of classifiers with cross-validation and plotting ROC curves [13] will prove the rationality of the experimental design method through experimental figures and tables with actual data and point out the conclusions and contributions of the paper

### 3.2. Dataset Analysis

Identify applicable sponsor/s here (*sponsors*).

First of all, it is necessary for preprocessing of the data. It is because the dataset comes from publicly available biological data and has undergone necessary sorting. However, in essence, it still requires witty preprocessing to determine appropriate inputs and outputs in order to make the experimental process more feasible and the experimental results more reliable.

  Dataset 1:
  Independent variable:
  Feature drug ID + clone ID + round measured + SLF34.1–173 as x_feature
  Dependent variable:
  Phenotype30 + reindexed as y_label
  Total data: (176 + 31) columns × 2701 rows = 559,107
  Dataset 2:
  Independent variable:
  Feature drug ID + clone ID + within-phenotype adjusted distance to unperturbed + *z*-scored SLF34.1-117 as x_feature
  Dependent variable:
  Human-assigned class for unperturbed experiment as y_label (dependent variable)
  Total data: (120 + 1) columns × 2162 rows = 261,602
  There are 80% as the training dataset and 20% as the test dataset with a random split among the total dataset
  At the same time, different splits will be performed according to the following different cases

### 3.3. Model Designed

Secondly, three sets of different designs were used in the experiment. During this level of experimentation, many machine learning models will be applied, compared, and verified. Therefore, this project calls this stage the model level.

The three sets of experiments are as follows:

  Case 1:
  There are nine models composed of nine different traditional machine learning methods, with the same data input and the same data output. The data used are the original data after removing the empty set and a small part of the data that are too close to 0 in the dataset, and the accuracy of these models and the computing time are compared under the same hardware conditions.
  Case 2:
  Using the optimal model and its approximate methods, a total of three models improve, adjust, optimize, and are from another perspective. The receiver operating characteristic (ROC) curve is applied to verify the model's functionality more comprehensively and with reliability. Among them, accuracy, precision, recall, true positive rate (TPR), false positive rate (FPR), area under the curve (AUC), and so on, will be fully considered. Furthermore, the data used here are 33% of the total data randomly.
  Case 3:
  Propose a new method (meta-active learning (MAML)), establish a machine learning model, and compare the traditional optimal model once again from a new angle uncertainty estimation to evaluate the model optima. Further considering, in this verification process, in order to eliminate the influence of the data itself on the output, the output effect of the model is compared with random. Still, this case uses other different methods to split the dataset.

### 3.4. Meta-Active Learning (MAML) Designed

Active learning is a method used under the premise of a small number of data samples. Although the data requirements are small, more training and optimization attempts are needed to obtain a feasible model. In addition, it can output many process parameters. Therefore, metalearning is added to use these process parameters as training data directly.

The specific method is designed to randomly split sampling 100 sets of data from the dataset and divide them into ten even samples. For all sample data, first use optimized machine learning methods for training, for instance, a logistic model with a loss function. Then, during the training process, output and record the parameters, such as loss function and normalization, in the logistic model. This paper expresses it as *R*(*μ*), and the two normalization methods L1 and L2 are discussed. Usually, this training method could be derived from the following formula:

(1) $$\begin{array}{c} \text{opt}\left(\mu ;\theta \right)=\sum_{k=1}^{n}\text{loss}\left(y_{i},\nu \left(x_{i};\mu \right)\right)\;+\theta R\left(\mu \right), \end{array}$$

where *x* and *y* represent the feature and label, respectively [14]. In order to obtain the optimal solution of the objective function $\hat{\mu }=\arg\underset{\mu }{\min}\text{opt}\left(\mu ,\theta \right)$, it is often necessary to specify hyperparameter *θ*, and this parameter is used as the input in the meta-active learning model, for example, the above ten samples ${\tilde{\theta }}_{n}=\left\{\theta_{1},\theta_{2},\ldots ,\theta_{10}\right\}$. These parameters are obtained in different optimization processes of the data. Thus, meta-active learning can directly generate the initial value, enabling the logistics to quickly obtain a relatively good extreme point. For this reason, it considerably simplifies the training operation process and the required software and hardware resources.

Finally, the verification level is actually to verify different verification methods of the above model. These methods are the current mainstream methods to verify the optima of machine models. However, in order to ensure that each step of the machine verification process is more reliable and try to eliminate the influence of errors, this paper uses different methods in different verification steps.

## 4. Results and Analysis

This section provides a detailed analysis of the results and a brief discussion on level-1 experiment results' analysis, level-2 experiment results' analysis, and level-3 experiment results' analysis.

### 4.1. Level-1 Experiment Results' Analysis

Define abbreviations and acronyms the first time they are used in the text, even after being defined in the abstract. Abbreviations such as IEEE, SI, MKS, CGS, sc, dc, and rms do not have to be defined. Do not use abbreviations in the title or heads unless they are unavoidable.

(2) $$\begin{array}{c} \text{Accuracy}=\frac{\sqrt{\sum_{k=1}^{n}{\left(\text{predictions}-\text{labels}\right)}^{2}}}{n}. \end{array}$$

This paper chooses nine traditional methods to build nine models: elastic net (EN); Bayesian ridge regression (BRR); ridge regression (RR); logistic regression (LoR); KNN regression (KR); linear regression (LiR); gradient boosting for regression (GBR); random forest regression (RFR); random forest classifier (RFC). This point is shown in Table 1.

Among them, the accuracy of the logistic regression method is the best, and it is prominent among other algorithms. Under the premise of the same hardware conditions and data volume, the linear regression method shows the least calculation time; however, the accuracy is not better. By careful considerations, this paper still selects logistic regression as the optimal model in case 1, and after that, it enters case 2.

### 4.2. Level-2 Experiment Results' Analysis

In this group of experiments, there are two normalization methods in scikit-learn used to solve the overfitting problem and further optimize the model effect.

(3) $$\begin{array}{c} \omega =\left(y_{i},\nu \left(x_{i};\mu \right)\right), \end{array}$$

(4) $$\begin{array}{c} \text{loss}{\left(\omega \right)}_{L1}=P\times \text{loss}\left(\omega \right)+\sum_{k=1}^{n}\left|\omega_{j}\right|\left(k\geq 1\right), \end{array}$$

(5) $$\begin{array}{c} \text{loss}{\left(\omega \right)}_{L2}=P\times \text{loss}\left(\omega \right)+\sqrt{\sum_{k=1}^{n}{\left|\omega_{j}\right|}^{2}}\left(k\geq 1\right). \end{array}$$

loss(*ω*) is the loss function, *P* is the hyperparameter used to control the degree of regularization, *n* is the total number of features in the equation and also the total number of parameters in the equation, and *k* represents each parameter. *k* must be greater than or equal to 1 because the first parameter in the parameter vector is the intercept *ω*_0_, which usually does not participate in normalization. Thus, OvA (one vs. all) treats all situations as binary logistic regression. At the same time, multinomial refers to the many-vs-many (MvM) situation.

It can be observed from Figure 3 and Table 2 that the method accuracy of L1 logistic is higher. Therefore, it is better than the other two logistic methods. Due to the huge amount of original data and 51 classes, to compare the three logistic methods more clearly, the first three and the first five classes are selected, shown in the classification probabilities in the figure. The classification probability means the probability of a certain data point belonging to each category, and an inverse heat map further represents it. In the figure, white “o” represents the training data. The more concentrated the centre of the image, the higher the correlation between its class and the accuracy of the result. In addition, the lighter the colour in the image, the higher the probability. Therefore, the lighter the overall colour is and the closer white “o” is to the class in the centre of the image, the stronger the effect is in the result. After selecting L1 logistic as the optimal model in case 2 and determining that L1 is the optimal loss function, enter Case 3.

### 4.3. Level-3 Experiment Results' Analysis

In MAML design, this project has described the method design process in Section 3 in detail. So, here, the specific results of the level-3 experiment are shown in Figures 4 and 5.

This part of the calculation method uses the mainstream method of the ROC and related calculation formulas [15]. It can be clearly observed from the figure that the ROC curve rises slowly in the L1 logistic method in an iterative manner. When the best effect is achieved, the AUC of the mean ROC for six folds is 0.90 ± 0.02. In contrast, the meta-active learning method directly generates a better initial value of the hyperparameter *θ* and quickly obtains the optimal extreme point. The model can quickly find the optimal solution, and the AUC of the mean ROC of six folds is 0.98 ± 0.00.

In order to make the experiment more convincing, this paper changes the dimensions again to discuss the optimality of the experimental model. Specifically, by discussing the estimate uncertainty of meta-active learning and comparing it with L1 logistics and random sample, the experimental results are given in Figure 6 and Table 3.

This paper selects the mean + standard deviation method and again randomly selects 100 numbers of queries. It is evident from the figure that initially, at the stage with fewer numbers of queries (≤40), the L1 logistic method is slightly better than others in some cases. In the meta-active learning estimate uncertainty method, it is difficult to establish an effective model because there are too few inputs for meta-active learning. In the stage with more numbers of queries (>40), meta-active learning has played an advantageous role. Its performance began to increase rapidly and remained around 0.95. In contrast, the L1 logistic method can only remain around 0.85, and its superiority to the random sample has become less and less noticeable. On the contrary, it can be observed from the table that the average performance of the meta-active learning estimate uncertainty is still higher than that of the L1 logistic. At the same time, the random sample is the lowest. Therefore, the performance of the model can also be observed as the performance at the level of the average values.

## 5. Conclusion

In this application scenario on biological data-driven experimentation, this article first uses nine machine learning models to filter out the optimal model. They effectively solve data problems that other models cannot handle. This model is further optimized to improve its accuracy. This paper designed a meta-active learning model for solving the problem of manually labeling a smaller number of labels. This model can meet the above accuracy and perform machine learning on the machine learning modelling process parameters. It has less calculation and accuracy than other models, the retention effect is stronger, and the experimental conclusion proves this theory.

The completed experiment results are used as the model of the next experiment, and further improvements and optimization are carried out. Each experiment is verified from multiple angles through different verification methods. For example, the level-1 experiment is to compare nine traditional machine learning methods. This paper uses accuracy and time as the criteria for judging the optimal model. The level-2 experiment discusses the comprehensive distribution of accuracy probability; the level-3 experiment uses the comprehensive judgment of performance and ROC.

The main contribution of this project starts from the conventional method, which most scholars are accustomed to choosing to face a data scenario, and research it step by step in depth. After that, it was obtained from each level of the experiment and related graphs through the analysis and discussion of the results. In a nutshell, this paper gets the best model and summarizes the most suitable method for processing this type of data. Furthermore, it designs feasible and reasonable methods for such scenarios. It provides reference and inspiration for solving similar scenarios and data problems.

## Figures and Tables

**Figure 1:** Concept graph of introduction.

**Figure 2:** Overview of modelling comparison.

**Figure 3:** Level-2 experiment results with probability.

**Figure 4:** Receiver operating characteristic results of L1 logistic.

**Figure 5:** Receiver operating characteristic results of metalearning.

**Figure 6:** Level-3 experiment results with meta-active learning estimate uncertainty.

**Table 1:** Level-1 experiment results with time.

Table head	EN	BRR	RR	LoR	KR	LiR	GBR	RFR	RFC
Accuracy (%)	0.93	0.92	0.92	0.96	0.93	0.92	0.92	0.92	0.91
Time (seconds)	0.998	0.010	0.022	0.803	0.025	0.001	5.623	3.190	0.024

**Table 2:** Level-2 experiment results with probability.

Methods	Accuracy (%)
Logistic regression with L1	75.0
Logistic regression (multinomial) with L2	74.4
Logistic regression (OvA) with L2	73.4

**Table 3:** Level-3 experiment results with meta-active learning estimate uncertainty.

Methods	Number_of_queries	Number_of_different_splits	Performance	Batch_size
Query instance uncertainty	100	10	0.904 ± 0.06	1
Query L1 logistic	100	10	0.817 ± 0.04	1
Query random	100	10	0.656 ± 0.05	1

## Data Availability

The data used to support the findings of this study are included within the article.
